# Disulfiram Suppresses Growth of the Malignant Pleural Mesothelioma Cells in Part by Inducing Apoptosis

**DOI:** 10.1371/journal.pone.0093711

**Published:** 2014-04-01

**Authors:** Vino T. Cheriyan, Ying Wang, Magesh Muthu, Shazia Jamal, Di Chen, Huanjie Yang, Lisa A. Polin, Adi L. Tarca, Harvey I. Pass, Q. Ping Dou, Sunita Sharma, Anil Wali, Arun K. Rishi

**Affiliations:** 1 Barbara Ann Karmanos Cancer Institute, Detroit, Michigan, United States of America; 2 Department of Oncology, Wayne State University, Detroit, Michigan, United States of America; 3 Department of Computer Science, Wayne State University, Detroit, Michigan, United States of America; 4 John D. Dingell VA Medical Center, Detroit, Michigan, United States of America; 5 Division of Cardiothoracic Surgery, New York University Cancer Center, New York, New York, United States of America; 6 Department of Life Science and Engineering, Harbin Institute of Technology, Harbin, China; University of Kansas Medical Center, United States of America

## Abstract

Dithiocarbamate compound Disulfiram (DSF) that binds with copper and functions as an inhibitor of aldehyde dehydrogenase is a Food and Drug Administration approved agent for treatment of alcoholism. Copper complexed DSF (DSF-Cu) also possesses anti-tumor and chemosensitizing properties; however, its molecular mechanisms of action remain unclear. Here we investigated malignant pleural mesothelioma (MPM) suppressive effects of DSF-Cu and the molecular mechanisms involved. DSF-Cu inhibited growth of the murine as well as human MPM cells in part by increasing levels of ubiquitinated proteins. DSF-Cu exposure stimulated apoptosis in MPM cells that involved activation of stress-activated protein kinases (SAPKs) p38 and JNK1/2, caspase-3, and cleavage of poly-(ADP-ribose)-polymerase, as well as increased expression of sulfatase 1 and apoptosis transducing CARP-1/CCAR1 protein. Gene-array based analyses revealed that DSF-Cu suppressed cell growth and metastasis-promoting genes including matrix metallopeptidase 3 and 10. DSF inhibited MPM cell growth and survival by upregulating cell cycle inhibitor p27Kip1, IGFBP7, and inhibitors of NF-κB such as ABIN 1 and 2 and Inhibitory κB (IκB)α and β proteins. DSF-Cu promoted cleavage of vimentin, as well as serine-phosphorylation and lysine-63 linked ubiquitination of podoplanin. Administration of 50 mg/kg DSF-Cu by daily i.p injections inhibited growth of murine MPM cell-derived tumors *in vivo*. Although podoplanin expression often correlates with metastatic disease and poor prognosis, phosphorylation of serines in cytoplasmic domain of podoplanin has recently been shown to interfere with cellular motility and migration signaling. Post-translational modification of podoplanin and cleavage of vimentin by DSF-Cu underscore a metastasis inhibitory property of this agent and together with our *in vivo* studies underscore its potential as an anti-MPM agent.

## Introduction

Malignant pleural mesothelioma (MPM) is an aggressive malignancy that is associated with past asbestos exposure. Millions of workers in the US and world over have been exposed to asbestos, and exposure to asbestos has been shown to increase the risk of several serious diseases including asbestosis, lung cancer and MPM [1]. It is estimated that there are 2,000 to 3,000 people diagnosed with MPM each year in the United States and the incidence of this disease is expected to increase in the next decade in United States and Europe [3], [4]. MPM is a rapidly progressing thoracic cancer that is characterized with late metastases and poor prognosis [1]. MPM is highly resistant to conventional therapies that consist of multimodality treatment involving surgery, adjuvant or neoadjuvant chemotherapy, and radiation [2]. The median survival of MPM is about 9–17 months [3], and coupled with its increasing incidence and resistance to currently available chemotherapies, development of new treatments for MPM is urgently needed.

Disulfiram (DSF) is a member of the dithiocarbamate family comprising a broad class of molecules possessing an R1R2NC(S)SR3 functional group, which gives them the ability to complex metals and react with sulfhydryl groups [5]–[7]. DSF, an irreversible inhibitor of aldehyde dehydrogenase, is one of the two drugs approved by the Food and Drug Administration (FDA) for treatment of alcoholism [7]. Clinical trials have shown efficacy of DSF with minimal to absent toxicity [7]. Several studies have shown that DSF and its metabolites can potentiate the effects of some anticancer drugs [8], [9]. Previous studies have demonstrated that DSF is capable of binding copper and forms a new complex (DSF-Cu). A number of recent studies have further highlighted a requirement of copper in DSF-induced toxicity and radiosensitization of cancer cells, induction of oxidative stress, and inhibition of NF-κB and proteasome by DSF-Cu in a variety of cancer cell types. However, the precise molecular mechanisms of DSF-Cu actions remain to be elucidated [10]–[13].

Here we investigated the MPM inhibitory properties of DSF-Cu and the molecular mechanisms involved. Although DSF-Cu stimulated activation of pro-apoptotic SAPKs, and caspase-9, -3, our gene-array-based analysis revealed that DSF-Cu suppressed expression of cell growth and metastasis transducers such as matrix metallopeptidase 3 and 10. Moreover, DSF-Cu suppression of MPM cell growth involved stimulation of a novel transducer of cell growth and apoptosis signaling CARP-1/CCAR1 [14]–[16]. Intra-peritoneal administration of DSF-Cu suppressed growth of murine mesothelioma allografts in part by enhancing apoptosis. Our proof-of-concept studies reveal, for the first time, MPM inhibitory properties of DSF-Cu and are expected to facilitate utilization of this agent or its potent derivatives as potential adjuvant for treatment and perhaps chemoprevention of MPM.

## Materials and Methods

### Cells and Reagents

Human MPM cell lines (H2373, H2452, H2595, H2714 and H2461) were previously established in our laboratory and characterized in detail as described elsewhere [17]. The MPM cells were cultured in either RPMI 1640 or DMEM-F12 supplemented with 100units/ml of penicillin, 100 µg/ml streptomycin, 4 mM L-glutamine, and 10% fetal calf serum. H226 and H-Meso MPM cells were obtained from ATCC (Manassas, VA) and maintained following vendor's guidelines. The murine MPM AB12 cell line was derived from BALB/c mice and was previously shown to form subcutaneous tumors when implanted in mice [18], [19]. AB12 cells were cultured and maintained in high-glucose DMEM supplemented with 10% fetal bovine serum (FBS), 100 units/mL penicillin, 100 µg/mL streptomycin. Cells were incubated at 37°C in a humidified atmosphere of 5% CO2 in air and were passaged weekly.

Fetal bovine serum (FBS) was obtained from Tissue Culture Biologicals (Tulare, CA). RPMI 1640 medium, penicillin and streptomycin were purchased from Invitrogen Co. (Carlsbad, CA). DMEM was purchased from Mediatech Inc (Herndon, VA). DSF, CuCl_2_, dimethyl sulfoxide (DMSO), anti-β-actin mouse monoclonal antibody, and 3–4, 5-dimethyltiazol-2-yl-2.5-diphenyl-tetrazolium bromide (MTT) were purchased from Sigma-Aldrich (St. Louis, MO). A 50 mM stock of DSF-copper mixture was prepared in DMSO as described before [20] and stored at −20°C. Mouse monoclonal antibody p21 and the caspase-3/-7-specific substrate Ac-DEVD-AMC were obtained from Calbiochem Inc. (San Diego, CA). Anti-PARP mouse monoclonal antibody was purchased from BIOMOL International LP (Plymouth Meeting, PA). Anti-ABIN2, vimentin, c-myc (9E10), and Ubiquitin (p4D1) monoclonal antibodies and anti-p27 (F-8) polyclonal antibodies were purchased from Santa Cruz Biotechnology Inc. (Santa Cruz, CA). Mouse monoclonal antibody NCL-p27 was purchased from Novocastra Laboratories Ltd (Newcastle upon Tyne, UK). Anti-p38, phospho-p38, PARP, ABIN1, IκBα, and IκBβ rabbit polyclonal antibodies, caspase-3, and phospho-JNK (threonine183/tyrosine 185) G9 mouse monoclonal antibodies were obtained from Cell Signaling Technology (Beverly, MA). The phospho-serine monoclonal antibody 16B4 that specifically recognizes phosphorylated serine residues that are immediately followed by lysine (pSK, substrate for CDC kinase) or proline (pSP, substrate for MAP/SAP kinases) was obtained from Enzo Life Sciences (Farmingdale, NY) while anti-Ubiquitin, Lys63-Specific (Clone Apu3) and Anti-Ubiquitin, Lys48-Specific, (Clone Apu2) rabbit monoclonal antibodies were obtained from Millipore (Temecula, CA). Anti-podoplanin D2-40 mouse monoclonal (SIG-3730; antigen M2A) and rat monoclonal {Clone NZ-1.2; antigen: synthetic peptide corresponding to amino acids 38–51 (EGGVAMPGAEDDVV) of podoplanin} were purchased from Covance (Dedham, MA) and Imgenex (San Diego, CA), respectively. Anti-HSulf-1 rabbit polyclonal antibodies were purchased from Abcam (Cambridge, MA). Anti-IGFBP7 polyclonal antibodies were purchased from R&D Systems, Minneapolis, MN. Generation and characterization of the anti-CARP-1/CCAR1 rabbit polyclonal antibodies have been described before [14]. Enhanced Chemiluminescence Reagent was purchased from Amersham Biosciences (Piscataway, NJ) and the Apoptag Peroxidase In Situ Apoptosis Detection Kit was obtained from Chemicon International, Inc. (Temecula, CA). Protein Assay Kit and ApoAlert Caspase profiling plate were purchased from Bio-Rad Laboratories (Hercules, CA) and Clontech (Mountain View, CA), respectively.

### Cell Growth Inhibition Studies by MTT Assay

MPM cells (5×10^3^) were seeded in a 96-well culture plate and subsequently treated with DSF-Cu at different concentrations for noted times. Control cells were treated with 0.1% DMSO in culture medium. After treatment, the cells were incubated with 1 mg/ml of MTT reagent at 37°C for 4 hours and then MTT was removed and 100 µL of DMSO was added, followed by colorimetric analysis using a multi-label plate reader at 560 nm (Victor3; PerkinElmer, Wellesley, MA, USA).

### Cell-Free Caspase Activity Assay

MPM cells were treated with different concentrations of DSF-Cu for indicated time periods. The prepared whole cell extract (30 µg per sample) was then incubated with 40 µM of caspase-3/-7 substrate Ac-DEVD-AMC in 100 µl of the assay buffer (20 mM Tris–HCl, pH 7.5) at 37°C for at least 2 h. The release of the AMC groups was measured as above. In addition, activation of caspases in DSF-Cu-treated MPM cells was measured by utilizing the ApoAlert Caspase profiling plate essentially as described before [21].

### Western Blot and Immuno-Precipitation Analysis

Logarithmically growing MPM cells were treated with DSF-Cu for indicated dose and times, harvested and lysed in RIPA buffer (50 mM Tris-HCI, pH 8.0, 150 mM sodium chloride, 1.0% NP-40, 0.5% sodium deoxycholate, 0.1% sodium dodecyl sulfate, and 0.1% of protease inhibitor cocktail) for 20 min at 4°C. The lysates were centrifuged at 14,000 rpm at 4°C for 15 min to remove debris. Protein concentrations of the clarified cell lysates were determined using the Protein Assay Kit (Biorad). Approximately 1 mg of protein from each of the untreated and DSF-treated cell lysates was subjected to immuno-precipitation in conjunction with anti-phospho-serine 16B4 monoclonal antibody, anti-lys48-linked ubiquitin antibody, or anti-lys63-linked ubiquitin antibody as described [16]. Supernatant proteins, 50 µg from each sample, or the immuno-precipitated complexes were separated by SDS-10% polyacrylamide gel electrophoresis (SDS-PAGE) and transferred to polyvinylidene difluoride (PVDF) membrane (Bio-rad, Hercules, CA) by standard procedures. The membranes were hybridized with primary antibodies followed by incubation with appropriate secondary antibodies. The antibody-bound proteins were visualized by utilizing the chemiluminescence detection reagent (Pierce) according to manufacturer's instructions, followed by exposure to Kodak X-Omat X-ray film (Sigma) or hyblot ES Autoradiography film (Denville Scientific, Inc., Metuchen, NJ). The membranes having protein extracts were re-probed with the anti-β actin antibody, which was used as an internal control for protein loading.

### Isolation of RNA and Microarray Analysis

The H2373 MPM cells were either untreated or treated with DSF-Cu (2.5 µM; 24 h), and cells were harvested and total RNA were isolated, and purified using the RNeasy Mini kit and RNase-free DNase Set (Qiagen, Valencia, CA) according to the manufacturer's protocols. DSF-Cu-dependent changes in gene expression were analyzed at the Genomic Core Facility, Karmanos Cancer Institute utilizing Illumina BeadChip Arrays essentially according to manufacturer's instruction (Illumina, San Diego, CA). Briefly, 0.5 µg total RNA was biotin-labeled and hybridized with BeadChips. The signal was detected with streptovadin-Cy3 according to manufacturer's instruction (Illumina). The imaging of the BeadChips was conducted using a Bead Array Reader in conjunction with Bead Studio software (Illumina). The data was normalized using a quantile based approach which transforms the raw data so that the resulting normalized expression values of each sample have the same distribution [22]. We next performed an unsupervised cluster analysis to detect similarities among samples based on gene expression profiles. The genes retained to perform the clustering were those varying the most regardless their group membership as described elsewhere [23]. Significance of the differentially expressed genes among control (untreated) and DSF-Cu-treated groups was determined using a moderated t-test. The corrected p-values were calculated by adjusting p-values using the False Discovery Rate method. The p values of <0.5 were considered significant provided that the fold change in expression was also equal to or larger than 1.5.

### Murine Mesothelioma Allograft Experiments

The experiments involving xenograft studies were performed in accordance with protocols approved by the Wayne State University Institutional Laboratory Animal Care and Use Committee (WSU-IACUC). Five week-old, female BALB/c mice were purchased from Taconic Research Animal Services and housed in accordance with WSU-IACUC protocols. On day 1 AB12 murine MPM cells (0.5×10^6^) were suspended in 0.1 mL serum-free DMEM medium and inoculated subcutaneously (s.c.) in the right flank of each mouse (n = 5 each group). On the day 10 following inoculation the tumors became palpable. At that time, the mice were randomly assigned into 2 groups. The control group animals received a daily i.p. injection with 50–100 µl of vehicle (PBS/cremophor/DMSO/ethanol, 7.5∶1.5∶0.5∶0.5) formulation. The test group animals on the other hand received 50–100 µl of the vehicle containing 50 mg/kg DSF-Cu daily. Tumor sizes were measured daily using calipers and their volumes calculated using a standard formula: width^2^×length/2. Body weight of the animals in the test and treatment groups were measured weekly. The mice were sacrificed after 16 day-treatment when control tumors reached to ∼1000 mm^3^. H&E staining of xenograft tissue was carried out to confirm presence of tumor.

### Immunohistochemical Analysis

Apoptosis in tumor tissues was determined by TUNEL assay using in situ cell Death Detection kit from Roche Applied Science (Indianapolis, IN) according to the manufacturer's instruction. The formalin-fixed tumor xenograft biopsies from the animals that were untreated or treated with DSF-Cu were paraffin embedded and processed essentially following our previously described procedures [24]. The tumor tissue slides were stained for presence of CARP-1 and cyclin-dependent kinase inhibitor p27 by utilizing respective antibodies, and were then photographed using Zeiss microscope with a 35 mm camera attached for recording the photomicrographs. H&E counter-staining of tumor tissues was performed following our previously described methods [24].

## Results

### DSF-Cu Inhibits MPM Cell Proliferation

In light of the emerging anti-cancer properties of DSF-Cu, we first determined whether this compound inhibits MPM cell growth in vitro. For this purpose, we utilized five human MPM cell lines. As shown in figure 1, DSF-Cu inhibited cell proliferation in all tested cell lines. A 1 µM dose of DSF-Cu elicited ∼70% loss of viability of all but H2595 MPM cells (Figure 1). H2595 cells were relatively less sensitive to DSF-Cu treatment, exhibiting ∼30% loss of viability at the 1 and 5 µM doses. Since the MPM cells utilized here are representative of the epitheliod (H2461 and H2595), sacromatoid (H2373), and biphasic (H2452) tumor histologic origins [17], [25], and the treatments with DSF-Cu significantly inhibited viabilities of most of these cells, the data would suggest for potential utility of this agent to target a diverse histotypes of MPM tumors.

**Figure 1:** DSF-Cu reduces viabilities of the human MPM cells. Cells were treated with vehicle (DMSO) or the indicated doses of DSF-Cu for noted time. Determination of viable/live cells was carried out by MTT assay. Data in the histogram represents means of three independent experiments; bars, S.E. *, p<0.05 relative to vehicle-treated H2373, H2461, H2452, and H2714 cells.

### DSF-Cu Promotes Protein Ubiquitination and Apoptosis in MPM Cells

We have previously noted that human breast cancer cell growth inhibition by DSF-Cu involved stimulation of apoptosis [20]. Consistent with these findings, treatments of H226, H-Meso, and AB12 mouse MPM cells with DSF-Cu resulted in morphological changes such as nuclear condensation and fragmentation associated with apoptosis in a dose-dependent manner (Figure 2A). To further confirm that apoptosis induction involved DNA fragmentation, AB12 murine MPM cells were directly cultured in a 4-well chamber slide and treated with DSF-Cu and immunocytochemical labeling of the fragmented DNA was carried out as detailed in methods. Treatment of murine MPM cells with DSF-Cu resulted in increased number of TUNEL-positive cells (Figure 2B). Since activation of caspases is a crucial step in transduction of apoptosis signaling, we next determined whether caspases were activated in MPM cells undergoing apoptosis following exposure to DSF-Cu. For this purpose, we profiled activation of caspases 2, 3, 8, and 9 in different MPM cells following their treatments with DSF-Cu utilizing a fluorescence-based quantitative assay as described in methods. As expected, DSF-Cu stimulated caspase-3 activation in a dose-dependent manner in H226, H-Meso and AB12 MPM cells (Figure 2C). In addition, a 1 µM dose of DSF-Cu stimulated a robust stimulation of caspases-3 and 9 but not caspases-2 or -8, in H2373 MPM cells (Figure 2D). Since caspase-8 and -9 are generally activated by extrinsic and intrinsic, mitochondria-mediated, apoptosis, respectively, and the activated caspases-8 and -9, in turn, activate down-stream effector caspase-3, activation of caspase-9 in MPM cells would suggest for an intrinsic, mitochondria-mediated, apoptosis signaling induced by this compound.

**Figure 2:** Apoptosis induction by DSF-Cu involves Caspase activation. (A) Indicated MPM cells were treated with different concentrations of DSF-Cu for 18 h. Photomicrographs showing apoptosis-associated morphological changes in MPM cells treated with DSF-Cu. 0, Control, DMSO treatment. (B) Murine MPM cells were either untreated (Control), or treated with DSF-Cu for noted dose and time. Staining of the cells was performed using TUNEL assay as detailed in Methods. Dark brown staining represents fragmented cell nuclei. (C) Indicated MPM cells were treated with DSF-Cu for noted time and concentrations, followed by analysis of caspase 3 activities by ELISA. DMSO was used as vehicle control. (D) MPM cells were either untreated (Control) or treated with DSF-Cu for indicated dose and time. Activities of the noted caspases were measured as in methods. Columns in histogram represent fold activation of respective caspases relative to the corresponding controls and were derived from means of two independent experiments.

Given that Bortezomib is the first proteasome inhibitor that has been approved in the US for treatment of relapsed multiple myeloma and mantle cell lymphoma, and a number of studies have revealed a proteasome inhibitory activity of DSF-Cu in breast cancer cells [20], [26], we next tested whether DSF-Cu exposure caused inhibition of proteasome in MPM cells. Since cellular proteasome system is designed to degrade proteins that have been tagged by ubiquitin moieties, especially the proteins that have lysine-48 linked polyubiquitination, we determined whether DSF-Cu treatments promoted ubiquitination of MPM cell proteins. Western immunoblot analysis revealed elevated ubiquitination of proteins in different MPM cells in the presence of DSF-Cu in a dose-dependent manner (Figure 3). Consistent with the fact that inhibition of proteasome often results in apoptosis induction, DSF-Cu exposure also promoted PARP1 cleavage in a dose-dependent manner in different MPM cells (Figure 3A). Together with the data in figure 2, these findings suggest that DSF-Cu suppresses MPM cell growth in part by inhibiting proteasome and activating intrinsic apoptosis signaling involving caspases 9 and 3.

**Figure 3:** DSF-Cu inhibits proteasome activity and induces apoptosis in MPM cells. Indicated MPM cells were treated with noted doses of DSF-Cu followed by western blot analysis for presence of ubiquitinated proteins and cleaved PARP (A), K-48 linked ubiquitinated proteins and p27Kip1 (B), and K-63 linked ubiquitinated proteins (C). The respective membranes were subsequently probed for levels of actin to confirm equal loading. Please note that DMSO was used as vehicle control (indicated as 0) for all the panels, while the DSF-Cu treatments in panel A were carried out for 18 h.

### DSF-Cu Suppression of MPM Cell Growth Involves Activation of Novel Apoptosis Signaling Pathways

Apoptosis stimulation by DSF-Cu has previously been shown to involve elevated levels of reactive oxygen species (ROS) in thymocytes, melanoma, and breast cancer cells [11], [27], [28]. Moreover, since intracellular levels of ROS are known to activate MAPKs/SAPKs signaling to regulate cell survival by modulating downstream pathways such as NF-κB signaling [29]–[31], we then investigated whether DSF-Cu exposure activated JNK and p38 SAPKs. Consistent with the findings in other cell models, our data show that DSF-Cu stimulated activation of JNK1/2 and p38α/β in a dose dependent manner in both the murine and human MPM cells (Figure 4). Infact, both the SAPKs were robustly activated in the MPM cells exposed to 1 µM or higher doses of DSF-Cu.

**Figure 4:** DSF-Cu activates pro-apoptotic SAPKs in MPM cells. MPM cells were either untreated (Control; noted as 0) or treated with indicated doses of DSF-Cu for noted time. Levels of phosphorylated JNK1/2 (noted as p-JNK1) and actin protein (A, B), or p38α/β (noted as p-p38), and total p38 proteins (C, D) were determined by Western blotting essentially as in figure 3.

To further elucidate the molecular mechanisms of MPM cell growth inhibition by DSF-Cu, gene-array-based high throughput analysis was carried out. Human MPM cells were either untreated or treated with DSF-Cu and respective cellular RNAs were isolated and utilized to synthesize labelled, first strand cDNAs as detailed in methods. The labelled first strand cDNAs from each group were separately hybridized with Illumina gene-array chips, and data were analyzed to identify mRNAs that had a significant, 1.5-fold or higher altered expression in the MPM cells that were treated with DSF-Cu essentially following the procedures noted in methods and our previously published studies [21], [32]–[34]. A select subset of genes that were either up-regulated or down-regulated in MPM cells exposed to DSF-Cu are presented in table 1 (please refer to table S1 for a complete list of MPM genes that were modulated by DSF-Cu). The array-data revealed that DSF-Cu treatment caused down-regulation of a large number of genes that were generally associated with cell growth and survival signaling, while a small group of cell growth inhibition/apoptosis-signaling genes were up-regulated following treatment of MPM cells with DSF-Cu. The group of genes that were down-regulated following treatments of MPM cells with DSF-Cu included transcription factors such as Forkhead box J1 and A3, FosB and cFos, early growth response (EGR)1, deacetylases (SIRT1 and SIRT6), Heparin-binding Epidermal growth Factor-like growth factor (HBEGF), and cell growth and metastasis-promoting genes such as ras-related C3 botulinum toxin substrate 1 (small GTP binding protein p21Rac1), matrix metalloproteinase (MMP) 3 and 10 (Table 1). A small subset of genes that were up-regulated following treatment of MPM cells with DSF-Cu included Insulin-like growth factor binding protein (IGFBP)7, growth arrest-specific (GAS)6, SMAD3, and sulfatase (SULF)1. Of note is the fact that a robust, ∼8.0-fold increase in the expression of IGFBP7 was noted in the MPM cells that were treated with DSF-Cu (Table 1). IGFBP7 signaling are often associated with cell growth suppression [35], and elevated expression of SULF1 has also been shown to inhibit HBEGF-dependent co-receptor functions of cell surface heparan sulfate proteoglycans (HSPGs) in hepatic and esophageal squamous cell cancer cells [36], [37]. We next determined whether DSF-Cu treatments stimulated SULF1 and IGFBP7 expression in MPM cells. An increase in SULF1 and IGFBP7 levels was noted in the human MPM cells following their treatments with DSF-Cu in a dose-dependent manner (Figure 5B). Therefore, it is likely that stimulation of IGFBP7 and SULF1 signaling coupled with attenuation of survival signaling due in part to the reduced levels of HBEGF, EGR1, SIRT1/6, and FosB/cFos proteins function to inhibit MPM cell growth in the presence of DSF-Cu.

**Figure 5:** DSF-Cu enhances expression of cyclin-dependent kinase inhibitor p27Kip1, and pro-apoptotic CARP-1, IGFBP7, and Sulfatase1 proteins. Murine (A) or human (B) MPM cells were either untreated (Control; noted as 0) or treated with indicated doses of DSF-Cu for noted time. Cell lysates were analyzed by Western blotting for levels of CARP-1, Sulfatase1, p27Kip1, IGFBP7, and actin proteins as in Methods.

**Table 1:** List of select genes regulated by DSF-Cu in MPM cells.

Symbol	Name	REFSEQ	Adjusted p-Value	Fold Change	Direction
BTK	Bruton agammaglobulinemia tyrosine kinase	NM_000061.2	3.97043E-07	1.86	DOWN
FOXJ1	Forkhead box J1	NM_001454.3	5.52166E-05	1.6	DOWN
SIRT1	Sirtuin (silent mating type information regulation 2 homolog) 1 (S. cerevisiae)	NM_001142498.1	0.018	2.36	DOWN
SNAI1	Snail homolog 1 (Drosophila)	NM_005985.3	0.023	8	DOWN
FOXA3	Forkhead box A3	NM_004497.2	0.039	1.88	DOWN
MAP3K13	mitogen-activated protein kinase kinase kinase 13	NM_001242314.1	0.041	1.4	DOWN
FOSB	FBJ murine osteosarcoma viral oncogene homolog B	NM_001114171.1	0.052	5.8	DOWN
MMP10	Matrix Metallopeptidase 10 (stromelysin 2)	NM_002425.2	0.055	3.29	DOWN
SIRT6	Sirtuin (silent mating type information regulation 2 homolog) 6 (S. cerevisiae)	NM_001193285.1	0.077	1.48	DOWN
IGFBP7	Insulin-like growth factor binding protein 7	NM_001253835.1	0.243	8.19	UP
GADD45B	Growth Arrest and DNA-damage-inducible, beta	NM_015675.3	0.389	6.56	DOWN
FOS	v-fos FBJ murine osteosarcoma viral oncogene homolog	NM_005252.3	0.69	8.58	DOWN
IGF2R	Insulin-like growth factor 2 receptor	NM_000876.2	0.979	2.3	UP
SMAD3	SMAD family member 3	NM_001145102.1	0.989	2	UP
VGF	VGF nerve growth factor inducible	NM_003378.3	0.999	3	DOWN
EGR1	Early growth response 1	NM_001964.2	0.999	3	DOWN
BAG3	BCL2-associated athanogene 3	NM_004281.3	0.999	2.9	DOWN
HRK	Harakiri, BCL2 interacting protein (contains only BH3 domain)	NM_003806.2	0.999	2.4	DOWN
SLFN11	Schlafen family member 11	NM_001104587.1	0.999	2.8	DOWN
RAC1	Ras-related C3 botulinum toxin substrate 1 (rho family, small GTP binding protein Rac1)	NM_006908.4	0.999	4.5	DOWN
HBEGF	Heparin-binding EGF-like growth factor	NM_001945.2	0.999	2.2	DOWN
CXCR4	Chemokine (C-X-C motif) receptor 4	NM_001008540.1	0.999	2.15	DOWN
DDIT3	DNA-damage-inducible transcript 3	NM_001195053.1	0.999	2.54	DOWN
BDNF	Brain-derived Neurotrophic factor	NM_001143805.1	0.999	2.18	UP
JAG2	Jagged 2	NM_002226.4	0.999	2.3	UP
GAS6	Growth arrest-specific 6	NM_001143946.1	0.999	2.5	UP
MMP3	Matrix Metallopeptidase 3 (stromelysin 1, progelatinase)	NM_002427.3	0.999	3.5	DOWN
SULF1	Sulfatase 1	NM_001128204.1	0.999	2.46	UP

We have previously identified CARP-1/CCAR1 that functions as a novel transducer of cell growth inhibitory and/or apoptosis signaling by a variety of agents including DNA damaging chemotherapeutics Adriamycin (Doxorubicin) and etoposide [14]. The DNA damage signaling by CARP-1 was also found to require co-activation of tumor suppressor p53 [38]. Our recent studies further revealed CARP-1 induction in MPM cells following their treatments with proteasome inhibitor velcade [32], dietary agent curcumin [33], and a medicinal plant-derived compound withaferin A [34]. Since CARP-1 is a key transducer of cell growth inhibitory signaling by chemotherapy, and elevated levels of CARP-1 were noted in MPM cells that were treated with chemotherapeutic (velcade) and dietary/medicinal agents (curcumin and withaferin A), we determined whether DSF-Cu also induced CARP-1 expression in MPM cells. The data revealed that DSF-Cu treatments not only induced expression of cyclin-dependent kinase inhibitor p27Kip1, it also caused increased expression of CARP-1 in a dose-dependent manner in both the murine and human MPM cells (Figure 5). Since deprivation of serum growth factors results in elevated CARP-1 levels [14], elevated levels of CARP-1 and p27Kip1 by DSF-Cu then would underscore for a cell-cycle inhibitory property of this compound. It should be noted however that increase in p27Kip1 levels occurred at the 100 nM dose of DSF-Cu in both the human and murine MPM cells, while a 0.5 µM and 2.5 µM doses of DSF-Cu caused elevated CARP-1 levels in human and murine MPM cells, respectively (Figure 5). Therefore, it is likely that p27Kip1 expression in the presence of lower doses of DSF-Cu would provoke MPM cell cycle arrest, and continued expression of p27Kip1 and stimulation of CARP-1 at higher doses of DSF-Cu further exacerbates cell cycle arrest, while elevated levels of CARP-1, SULF1, and activation of JNK/p38 SAPKs in the presence of higher doses of DSF-Cu concomitantly signal for apoptosis in MPM cells.

### DSF-Cu Inhibits NF-κB Signaling in MPM Cells

The transcription factor NF-κB is an important anti-apoptotic and chemoresistance-related transcription factor that is activated by a range of extrinsic and intrinsic cellular signaling, and its activation is often associated with increased proliferation, growth and survival of cancer cells and poor prognosis in many cancers [39]. Although a number of studies have attempted to develop inhibitors of NF-κB and its signaling transducers, and many chemotherapeutic agents often function in part by blocking NF-κB signaling, inhibition of this versatile transcription factor and its signaling nonetheless remain an attractive and desirable attribute for development of novel anti-cancer strategies [40]. Exposure of glioblastoma and breast cancer cells to DSF-Cu has previously been shown to attenuate transcriptional activation functions of NF-κB [11], [12], [31]. We next determined whether DSF-Cu also impacted activation of NF-κB in MPM cells. NF-κB activities are often regulated by its upstream kinase known as Inhibitory κB Kinase (IKK), and activated IKK phosphorylates IκBα/β, the endogenous inhibitors of NF-κB. The phosphorylated IκBα/β, in turn, are ubiquitinated and degraded by proteasome, allowing NF-κB nuclear translocation and transcriptional activation functions [39]. Moreover, signal and context-dependent regulation of IKK activation by upstream kinases and/or inhibitory molecules such as A20 binding inhibitor of NF-κB (ABIN) 1 and 2 proteins are also known to regulate NF-κB activities. Our WB analysis of cell lysates derived from MPM cells treated with DSF-Cu revealed elevated levels of IκBα and β proteins (Figure 6). DSF-Cu caused increased expression of IκBα and β proteins in a dose-dependent manner in both the murine and human MPM cells (Figure 6). In addition, DSF-Cu treatments also caused increased expression of ABIN1 and 2 proteins in a dose-dependent manner in both the MPM cell lines (Figure 6). Since ABINs are negative regulators of IKK, and are known to impact canonical NF-κB signaling, and the fact that IκBα and β are key inhibitors of both the canonical and atypical NF-κB signaling [41], the data in figure 6 suggest that DSF-Cu treatments block two central pathways of NF-κB activation in MPM cells.

**Figure 6:** DSF-Cu inhibits both the canonical and atypical NF-κB signaling. AB12 (A) and H2373 (B) MPM cells were either untreated (Control, noted as 0) or treated with indicated doses of DSF-Cu for noted time. Cell lysates were analyzed by Western blotting for levels of ABIN1, ABIN2, IκBα, IκBβ, and actin proteins as in Methods.

### DSF-Cu Inhibits MPM Cell Motility and Invasion Signaling and Inhibits Tumor Growth in Mesothelioma Allograft

Recent studies revealed that DSF-Cu inhibited clonogenicity of the breast cancer cells, and reduced neurosphere formation by the neuroblastoma and stem-like glioblastoma multiforme (GBM) cells [10], [31], suggesting that in addition to diminishing growth and proliferation, DSF-Cu treatments also attenuate the biological properties of the cancer cells. The biological properties of motility and invasion by the cancer cells are often regulated by a complex interplay of signaling by cell surface and intracellular proteins as well as the components of the extracellular matrix. A cell surface transmembrane glycoprotein, podoplanin, has been shown to regulate migration, epithelial-to-mesenchymal transition (EMT), and metastasis of cancer cells, and its expression is often related to malignancy and poor outcome in MPM and many other cancers [42]–[44]. Additionally, vimentin, an intracellular type III intermediate filament cytoskeletal protein, that regulates signaling for cell adhesion and migration, is also frequently elevated in invasive cancers and associates with metastasis and poor prognosis [45], [46]. Since, anti-MPM intervention approaches involving targeting of podoplanin or vimentin have recently been proposed [47], [48], we first determined whether DSF-Cu treatments also altered levels of these proteins in MPM cells. Western immunoblot analysis revealed a robust cleavage of vimentin by 0.5 µM or higher doses of DSF-Cu in both the murine and human MPM cells (Figure 7A, B).

**Figure 7:** DSF-Cu elevates expression and serine phosphorylation of podoplanin. (A, B) Indicated MPM cells were either untreated (Control, noted as 0), or treated with indicated doses of DSF-Cu for noted time. Cell lysates were analyzed for levels of podoplanin, vimentin, and actin proteins by Western blotting essentially as in figure 4. H2373 cells were either untreated (Control) or treated with DSF-Cu for indicated dose and time. The cell lysates (1 mg of protein) were first subjected to immunoprecipitation using anti-phospho-serine (C), anti-Ubiquitin (lys48-specific; not shown), or anti-Ubiquitin (lys63-specific) antibodies (D) as in methods. The membranes with the immunoprecipitates were then probed with anti-podoplanin D2-40 antibody as in panel A.

Western immunoblot analysis in conjunction with anti-podoplanin D2-40 monoclonal antibody revealed elevated levels of podoplanin peptides of 75 kDa or higher sizes in the human MPM cells that were treated with 1.0 and 2.5 µM doses of DSF-Cu (Figure 7A). In murine MPM cells however, expression of a 75 kDa podoplanin peptide was induced following treatments with 0.1 µM or higher doses of DSF-Cu (Figure 7B). Although the podoplanin cDNA encodes a peptide of 162 aminoacids with an expected molecular mass of ∼18–20 kDa, post-translational modifications such as glycosylation have been thought to result in ∼50 kDa or higher sized podoplanin peptides. To ascertain the extent DSF-Cu treatments caused additional post-translational modifications of podoplanin to result in its peptides of 75 kDa and higher sizes, we first analyzed podoplanin expression in conjunction with a second anti-podoplanin rat monoclonal antibody NZ-1.2 in the human MPM cell lysates derived from treatment with 2.5 µM DSF-Cu. Both the D2-40 and NZ-1.2 antibodies showed a robust increase in a ∼100 kDa peptide in lysates derived from DSF-Cu-treated cells (Figure S1). These data suggest that DSF-Cu treatments likely cause further post-translational modifications of the MPM cell surface podoplanin protein that collectively result in podoplanin peptides of 75 kDa and higher sizes.

A recent report demonstrated PKA phosphorylation of the serines in the intracellular region of podoplanin that resulted in diminished cell motility and migration signaling by podoplanin [49]. In addition, our ongoing studies also revealed serine phosphorylation and Lysine63-linked ubiquitination of podoplanin in MPM cells following their treatments with CFM-4, a member of a novel class of apoptosis-inducing small molecule compounds [50]. On the basis of these studies, we next determined whether exposure to DSF-Cu also resulted in serine phosphorylation of the intracellular tail of podoplanin, and subsequent ubiquitination of the phosphorylated podoplanin. Since Lysine63-linked ubiquitination often prevents degradation of the target proteins by the proteasome, and the fact that DSF-Cu inhibits proteasome and was also found to elevate cellular levels of ubiquitinated proteins (see figure 3), it is likely that the DSF-Cu treatments stimulate phosphorylation of podoplanin to inhibit its signaling for cell motility, while the Lysine63-linked ubiquitination contributes to a persistent and elevated levels of inactive podoplanin. Indeed, western immunoblot analysis of immunoprecipitates containing serine phosphorylated proteins present in the lysates derived from MPM cells treated with DSF-Cu revealed serine phosphorylation of an ∼100 kDa podoplanin peptide (Figure 7C). A similar western immunoblot analysis of the immunoprecipitates enriched for Lysine63-linked ubiquitinated proteins also revealed for the presence of a ∼100 kDa, ubiquitinated podoplanin protein in the MPM cells that were treated with DSF-Cu (Figure 7D). Treatments with DSF-Cu however failed to cause Lysine48-linked ubiquitination of podoplanin in the MPM cells (not shown). Collectively, the data in figure 7 suggest that DSF-Cu treatments likely interfere with motility and invasion properties of MPM cells in part by post-translational modifications of podoplanin and cleavage of vimentin proteins in the MPM cells.

To investigate whether DSF-Cu inhibits MPM tumor growth, we implanted murine mesothelioma AB12 cells (0.5×10^6^) subcutaneously into the right flanks of female Balb/c mice. When the tumors became palpable (∼120 mm^3^), mice were randomized into the 2 groups for treatment with vehicle control or DSF-Cu as detailed in methods. A daily dose of 50 mg/kg of DSF-Cu was administered i.p. for a 17-day period. Inhibition of tumor growth by DSF-Cu was observed after a 17 day–treatment, indicating the efficacy of DSF-Cu against mesothelioma (Figure 8A). After 17 days treatment, control tumors grew to an average size of 1786 mm^3^, and DSF-Cu–treated tumors grew to 509 mm^3^, corresponding to a 71% inhibition (Figure 8B). Tumor weights were measured by the end of the experiment. The average of tumor weight in vehicle treated group was 1.35 g, while it was 0.33 g in DSF-Cu-treated group, showing a 75% reduction in tumor weight (data not shown).

**Figure 8:** DSF-Cu inhibits murine MPM allograft growth. Female BALB/c mice bearing AB12 tumors were treated with either vehicle (Control) or DSF-Cu as described in methods. Animals were monitored every day for tumor volumes (growth) as well as any adverse effects. Tumor volumes and weights were measured as noted in methods. (A) Four tumors from control and two tumors from treated groups are shown. (B) Histogram showing tumor volumes of the control and DSF-Cu-treated groups. Points, mean tumor volume in each experimental group; Bars, SE. (C) Formalin-fixed tumor xenograft biopsies from panel A were paraffin embedded, processed, and subjected to immuno-staining as described in methods. Representative photomicrographs (400× magnification) in the first, top row show hematoxylin and eosin (H&E) staining of the tissue sections. Representative photomicrographs (400× magnification) are also shown to indicate for apoptosis (by TUNEL assay; second row), levels of p27Kip1 (third row), and CARP-1 (fourth row) proteins as noted in methods.

We next determined whether DSF-Cu inhibited murine MPM tumor growth by promoting apoptosis and stimulating expression of p27Kip1 and CARP-1 proteins. Levels of apoptosis in the murine MPM tumors that were either untreated (control) or treated with DSF-Cu were determined using the TUNEL assay, as well as immunostaining the tumors tissues for levels of p27Kip1 and CARP-1 proteins. The TUNEL staining indicated an increase in the number of apoptotic cells in a representative tumor from mouse treated with DSF-Cu when compared with the corresponding vehicle-treated control (Figure 8C). Consistent with the in vitro data in figures 2 and 6, increased apoptosis, and elevated levels of p27Kip1 and CARP-1 was also evident in a representative tumor that was derived from a mouse treated with DSF-Cu (Figure 8C). Taken together, these data show that DSF-Cu causes regression of mesothelioma growth in vivo in part by stimulating apoptosis.

## Discussion

Disulfiram, a dithiocarbamate is an alchohol dehydrogenase (ALDH) inhibitor, and is a widely used anti-alcoholism drug in clinic. Available pre-clinical and clinical data indicate suitable pharmacokinetic profiles and low to absent toxicities of this agent in humans. A number of investigations spanning over the last two decades have also revealed anti-cancer properties of this agent when complexed with copper. In fact disulfiram has been shown to facilitate copper uptake in cancer cells [51]. DSF-Cu inhibition of cancer cell growth involves pleiotropic mechanisms that include proteasome inhibition [20], generation of reactive oxygen species, attenuation of NF-κB activities [9], [11] and stimulation of apoptosis. Recent studies have further highlighted radiosensitizing and resistance-reversing properties of DSF-Cu in neuroblastoma and triple-negative breast cancer (TNBC) cells, respectively [10], [12]. A high through-put screening of ∼3000 compounds that are FDA-approved drugs recently identified disulfiram as a potent inhibitor of the TNBC cells [13], while other studies also demonstrated its abilities to inhibit breast cancer and glioblastoma stem cell-like cells [11], [31]. Consistent with emerging anti-cancer potential of DSF-Cu, our current studies revealed that DSF-Cu inhibits growth of a number of MPM cells. Of note are our proof-of-concept findings that DSF-Cu effectively inhibited growth of the MPM cells that were derived from the three different clinical histotypes of this malignancy. Although, the H2595 cells that were derived from the epitheliod tumor were relatively less sensitive, DSF-Cu nonetheless was effective inhibitor of another cell line derived from the epitheliod tumor (H2461), as well as the cells derived from the sarcomatoid (H2373) and biphasic (H2452) tumors [17]. In agreement with DSF-Cu mechanisms of action in other cancer cell models, our studies also revealed that MPM cell growth suppression by DSF-Cu involved elevated levels of ubiquitinated cellular proteins (likely the consequence of the well-known proteasome inhibitory properties of DSF-Cu), activation of stress-activated kinases JNK1/2 and p38α/β, inhibition of NFκB signaling, and stimulation of apoptosis (Figure 9). In addition to the proteasome inhibitory properties of DSF-Cu, a recent study revealed that DSF-Cu also inhibited E3 ligase BCA2 [52], and together with our data in figure 3B, C showing different kinetics of lysine-48 linked versus lysine-63 linked polyubiquitinted proteins in MPM cells further underscores pleiotropic mechanism of action of this agent. Whether inhibition of E3 ligases such as BCA2 contributed to the overall elevated levels of ubiquitinated cellular proteins in the presence of DSF-Cu, and to the extent this compound also targeted additional E3 ligases and/or deubiquitinases to cause elevated levels of ubiquitinated cellular proteins including the lysine-63 linked podoplanin (Figure 7D) remains to be clarified.

**Figure 9:** Schematic of key MPM growth inhibitory mechanisms utilized by DSF-Cu.

In an attempt to further elucidate the MPM inhibitory mechanisms of DSF-Cu, a high-through-put gene-array-based analysis was carried out. The data from this experiment revealed down-regulation of a large number of cell growth and survival regulatory genes in MPM cells treated with DSF-Cu. This subset included genes such as FOXJ1, FOXA3, FOSB, cFOS, SIRT1, SIRT6, EGR1, p21RAC1, MMP3 and 10. Since many cancer cells including MPM cells and tumors often express elevated levels of various MMPs, and the expression of MMPs is associated with poor prognoses, decreased expression of MMP3 and 10 proteins in MPM cells treated with DSF-Cu would suggest for a MPM metastasis-inhibitory property of this agent. Further evidence of the metastasis inhibitory potential of this compound could be deduced from our data in figure 7 where DSF-Cu was found to impact the functions of vimentin and podoplanin, two key molecules that are well known to regulate cancer cells motility, migration, and invasion signaling. Given that expression of both the podoplanin and vimentin proteins are often associated with poor prognosis in MPM and other cancers, cleavage of vimentin and post-translational modifications of podoplanin (phosphorylation and lys63-linked ubiquitination), and together with reduced expression of MMP3 and 10 proteins, would collectively suggest for MPM invasion and metastasis inhibitory properties of DSF-Cu.

The gene-array experiments also revealed increased expression of IGFBP7 and SULF1 proteins in the MPM cells exposed to DSF-Cu. SULF1 is often repressed in cancer cells by epigenetic mechanisms, and its re-activation interferes with cancer cell growth, invasion, and migration signaling [36], [37]. The tumor suppressor functions of SULF1 involve inhibition of co-receptor functions of cellular heparin sulfate proteoglycans (HSPGs). Since HSPGs regulate signaling by multiple receptor tyrosine kinases (RTKs) in the presence of heparin-binding growth factors such as HB-EGF, VEGF, PDGF, HGF, and FGF, DSF-Cu stimulation of SULF1 likely attenuates a range of receptor signaling pathways in MPM cells. Although it remains to be clarified whether DSF-Cu exposure caused diminished activation of any of the RTKs in MPM cells, the fact that HBEGF expression was reduced in MPM cells treated with DSF-Cu (Table 1) would suggest that signaling by various RTKs was likely targeted by DSF-Cu to inhibit MPM cell growth.

IGFBP7 is a member of the IGFBP family of proteins that exhibits low affinity for insulin-like growth factor (IGF) but binds insulin with high affinity [53], [54]. IGFBP7-dependent tumor suppression involves induction of senescence and/or apoptosis signaling, and its expression in tumor cells is often regulated by DNA methylation, retinoic acid and transforming growth factor (TGF)β [35], [53], [55], [56]. Although TGFβ-Receptor I (also known as ALK1) and SMAD-1/-5 pathway has previously been found to activate IGFBP7 expression in glioblastoma vascular and tumor endothelial cells where IGFBP7 plays a pro-angiogenic role [57], whether upregulation of SMAD-3 following treatment of MPM cells with DSF-Cu (Table 1) also caused elevated expression of IGFBP7, and to the extent this signaling contributed to MPM cell growth inhibition/apoptosis in the presence of DSF-Cu is intriguing and remains to be clarified. IGFBP7 is a secretory protein that is increasingly associated with tumor inhibitory effects in colon and breast cancers. Recent studies have further indicated that IGFBP7 expression is repressed by methylation –dependent mechanisms in colon cancers [58] while its paralog KAZALD1 is often methylated and silenced in MPM [59]. Although IGFBP7 expression has previously been proposed as a serum biomarker for bladder cancers [60], whether methylation-dependent mechanisms also regulate IGFBP7 expression in MPM, and to the extent its serum levels could be a useful biomarker in MPM have yet to be addressed. DSF-Cu treatments however robustly stimulated expression of CARP-1 (Figure 5) in the MPM cells. It is to be noted however that DSF-Cu caused elevated levels of cell cycle inhibitory p27Kip1 at lower doses while the levels of CARP-1 and SULF1 proteins were induced in MPM cells treated with higher doses of DSF-Cu. These findings suggest that cell growth arrest likely precedes the apoptosis signaling in the MPM cells that were exposed to varying doses of DSF-Cu.

The fact that elevated expression of IGFBP7, SULF1, and CARP-1 was also noted in curcumin-treated MPM cells [33], it is likely that MPM inhibitory mechanisms are utilized by DSF-Cu overlap with curcumin. Although oral administration of 200 mg/kg DSF-Cu did not inhibit neuroblastoma cell-derived xenograft growth in mice, it was nonetheless effective inhibitor of the neuroblastoma xenograft growth when administered in combination with radiation or radionuclide therapy [10]. Our studies revealed that intra-peritoneal administration of DSF-Cu was effective in inhibiting murine MPM allograft growth. Whether DSF-Cu efficacy noted in our studies is dependent on the histo-type of the tumor cells utilized for xenograft studies, and to the extent constitution of DSF-Cu formulation and its route of administration contributed to its anti-MPM efficacy remains to be clarified. DSF-Cu however was effective in suppressing murine MPM allograft growth, in part by stimulating expression of CARP-1, p27Kip1 and apoptosis (figure 8). Taken together, our proof-of-concept studies further elaborate anti-cancer properties of DSF-Cu, and underscore MPM inhibitory potential of this compound.

## Supporting Information

Figure S1 **Podoplanin expression in H2373 MPM cells.** MPM cells were either untreated (Control) or treated with DSF-Cu for noted dose and time. Cell lysates (50 µg protein/lane) were electrophoresed on two, 10% SDS-PAGE gels and proteins transferred to nitrocellulose membranes as in methods. One of the membranes was probed with anti-podoplanin antibody NZ-1.2 (autoradiogram on the right) and the other membrane was probed with anti-podoplanin D2-40 antibody (autoradiogram on the left). Both the membranes were subsequently probed with anti-actin antibody to assess loading.
(TIF)

Table S1 **List of DSF-Cu-regulated genes in H2373 MPM cells (XLSX).**
(XLS)
